# HGF and TGFβ1 differently influenced Wwox regulatory function on Twist program for mesenchymal-epithelial transition in bone metastatic versus parental breast carcinoma cells

This article has been retracted.

**DOI:** 10.1186/s12943-015-0389-y

**Published:** 2015-06-04

**Authors:** Paola Bendinelli, Paola Maroni, Emanuela Matteucci, Maria Alfonsina Desiderio

**Affiliations:** Dipartimento di Scienze Biomediche per la Salute, Molecular Pathology Laboratory, Università degli Studi di Milano, Milano, Italy; Istituto Ortopedico Galeazzi, IRCCS, Milano, Italy

**Keywords:** Mesenchymal epithelial transition, Hepatocyte growth factor, Wwox, Twist, HIF-1

## Abstract

**Background:**

Much effort has been devoted to determining how metastatic cells and microenvironment reciprocally interact. However, the role of biological stimuli of microenvironment in controlling molecular events in bone metastasis from breast carcinoma for mesenchymal-epithelial transition (MET) is largely unknown. The purpose of the present paper was to clarify (1) the influence of hepatocyte-growth factor (HGF) and transforming growth factorβ1 (TGFβ1) on the phenotype of bone-metastatic 1833 and parental MDA-MB231 cells; (2) the hierarchic response of Twist and Snail controlled by Wwox co-factor, that might be critical for the control of 1833-adhesive properties via E-cadherin.

**Methods:**

We studied under HGF and TGFβ1 the gene profiles—responsible for epithelial-mesenchymal transition (EMT), versus the revertant MET phenotype—making the correspondence with 1833 morphology and the relation to HGF-dependent control of TGFβ1 signalling. In particular, the activation of Twist program and the underlying molecular mechanisms were investigated, considering the role of endogenous and exogenous Wwox with siRNAWWOX and the expression vector transfection, to clarify whether Twist affected E-cadherin transactivation through a network of transcription factors and regulators.

**Results:**

HGF and TGFβ1 oppositely affected the expression of Wwox in 1833 cells. Under HGF, endogenous Wwox decreased concomitant with Twist access to nuclei and its phosphorylation via PI3K/Akt pathway. Twist activated by HGF did not influence the gene profile through an E-box mechanism, but participated in the interplay of PPARγ/Ets1/NF-*k*B-transcription factors, triggering E-cadherin transactivation. Altogether, HGF conferred MET phenotype to 1833 cells, even if this was transient since followed by TGFβ1-signalling activation. TGFβ1 induced Snail in both the cell lines, with E-cadherin down-regulation only in 1833 cells because in MDA-MB231 cells E-cadherin was practically absent. Exogenous Wwox activated metastatic HIF-1, with Twist as co-factor.

**Conclusions:**

HGF and TGFβ1 of bone-metastasis microenvironment acted co-ordinately, influencing non redundant pathways regulated by Twist program or Snail-transcription factor, with reversible MET switch. This process implicated different roles for Wwox in the various steps of the metastatic process including colonization, with microenvironmental/exogenous Wwox that activated HIF-1, important for E-cadherin expression. Interfering with the Twist program by targeting the pre-metastatic niche stimuli could be an effective anti-bone metastasis therapy.

**Electronic supplementary material:**

The online version of this article (doi:10.1186/s12943-015-0389-y) contains supplementary material, which is available to authorized users.

## Background

 The disparate nature of stimuli in metastasis microenvironment determines epithelial-mesenchymal transition (EMT), or more likely the molecular events that influence the reversion to MET phenotype [1–4].

The stimuli of tumour microenvironment converge upon the limited set of transcription factors Twist, Snail, ZEB and hypoxia inducible factor-1 (HIF-1), which can drive common and non-redundant pathways [5–8]. The zinc-finger factors Snail1 and Slug, and the two-handed zinc factor ZEB1 mediate the repression of the prototypical-epithelial marker E-cadherin [9, 10]. The switch between E- and N-cadherin is a classical example of dynamic modulation of cell adhesion in cancer-related EMT [10, 11].

The engineered loss of the EMT transcription factors evidences the importance of MET in lung metastasis from breast cancer, identifying Id1 and 3 as fundamental genes, and transforming-growth factor β (TGFβ)-Id1 signalling that opposes Twist [12]. The reversible induction of Twist1 promotes the metastasis from squamous cell carcinoma [13]. Although EMT seems a transient process, present at least only at the invasive front of carcinomas, while MET being the driving force for metastatic colonization [7], the molecular regulators that promote MET transition, critical for the formation of bone metastasis from breast cancer, are scarcely investigated.

To successfully complete the metastatic cascade, carcinoma cells adopt plasticity towards the neighbouring neoplastic cells and microenvironment, both the extracellular matrix storing growth factors and the supportive cells [1, 5, 14, 15]. Homotipic and heterotipic interactions are regulated by cell-adhesion molecules including E-cadherin [16], and cancer-cell E-cadherin interacts with N-cadherin on stromal-osteogenic cells [17]. E-cadherin expression diminishes in 50 % of breast-ductal carcinoma, whereas in breast-lobular carcinoma E-cadherin is completely lost in 90 % of cases [18]. We have demonstrated high E-cadherin expression in bone metastasis both from human breast ductal carcinoma and from 1833-xenograft model [19]. The 1833-bone metastatic clone derives from MDA-MB231-breast carcinoma cells [20]. The blockade of DNA-methyltransferase activities with 5’-Azacytidine, reducing the expression of E-cadherin and of the oncosuppressor WW-domain containing oxidoreductase (Wwox), changes the organotropism of the 1833 cells towards lung [19], leading to suppose Wwox-E-cadherin interactive function in bone metastasis.

Loss of heterozigosity and hypermethylation of *WWOX* enhance breast tumorigenesis; WW domains are important for protein interaction, and a nuclear-localization signal is present between the first and second WW domains of Wwox [21]. By undergoing Tyr33 phosphorylation and relocation to the nuclei, Wwox receives and integrates cell-surface signals like TGFβ [22]. Nuclear Wwox may either enhance or inhibit transcription-factor activities [23], and the transient overexpression of Wwox suppresses the activity of transcription factors by cytosol sequestering [22, 24].

The present paper will focus upon the existence of a time-dependent influence of hepatocyte growth factor (HGF) on TGFβ1 signalling in bone metastatic cells, compared to parental cells, with the aim to clarify whether microenvironment stimuli of bone metastasis contributed to EMT-MET switch and its reversion through Twist and Snail hierarchic response. In this context, we deepened the involvement of Wwox in the cellular localization and function of Twist and Snail, also under HGF stimulation, by overexpressing and knocking-down *WWOX*. Of note, in bone metastatic cells the transcriptional network was evaluated, taking into consideration also the function of Twist as HIF-1-activity regulator, because of the possible critical role in mesenchymal-epithelial plasticity by affecting adhesive properties. To address our hypothesis, we studied whether HGF and TGFβ1 had opposite and/or coordinated effects in determining the gene profiles- characteristic of EMT and MET in MDA-MB231 and 1833 cells- also by triggering a Twist program in 1833 cells for E-cadherin induction.

The growth factors of the bone microenvironment seem to influence bone-metastasis phenotype [1, 2, 4, 25], but the underlying molecular mechanisms are largely unknown. Twist and Snail might activate or repress target genes by employing several direct or indirect mechanisms. Modes of action by Twist1-bhelix-loop-helix (HLH) include direct DNA binding to E-box sequences, and recruitment of co-activators or repressors, but the regulatory outcomes of Twist are also controlled by spatio-temporal expression, phosphorylation and cellular localization [26]. The increase in Twist expression in patients is associated with poor survival and metastasis, whereas knock-down of Twist1 reduces breast cancer metastasis to bone [27].

We observed that in 1833 cells, HGF reduced nuclear Wwox and activated a Twist program. Consistently, siRNAWWOX enhanced Twist-transactivating activity. Twist program seemed transiently responsible for MET through E-cadherin induction and down-regulation of EMT-gene profile. MDA-MB231 cells did not show E-cadherin, and TGFβ1 stressed their mesenchymal phenotype differently from HGF. In 1833 cells, HGF via AMPK contributed to the activation of TGFβ signalling pathway, with reversion to EMT. Oppositely, exogenous-Wwox overexpression activated HIF-1, involving Twist as co-factor, and reduced Twist-luciferase activity also in the presence of HGF.

## Results

### In 1833 cells HGF increased nuclear expression and phosphorylation of Twist1, associated with Wwox down-regulation, differing from TGFβ1

To clarify whether the phenotype of bone metastasis from breast cancer depended on Twist and Snail, we evaluated their expression and intracellular localization in response to HGF and TGFβ1, two typical stimuli of bone microenvironment [1, 2, 4, 25].

As shown in Fig. 1a, HGF rapidly and persistently enhanced Twist-protein level in nuclear extracts of 1833 cells, being ineffective on Snail, and pTwist1/Twist ratio increased between 1 and 8 h, returning thereafter to the starvation value. On the contrary, TGFβ1 in nuclei transiently enhanced Snail-protein level peaking at 4 h, while Twist and its phosphorylated form progressively decreased. The level of Wwox co-factor increased in the nuclei 1.8- to 2.6-fold between 1 and 4 h after TGFβ1, and doubled after 16-h HGF. Since nuclear Wwox might be phosphorylated [22], immunoblot with anti-phosphoWwox was performed, and we observed that phosphoWwox increased 16 h after HGF and 4 h after TGFβ1 (Fig. 1b).

**Fig. 1:** HGF and TGFβ1 differently affected Twist and Snail in 1833 cells. We show representative images of Western blots, performed with nuclear (**a** and **b**) and cytosol (**c**) protein extracts from treated cells, and all the experiments were repeated three times with similar results. The samples were run on gel, and were processed under the same experimental conditions. B23, a marker of the nuclear fraction, and vinculin, a cytosolic protein, were used for normalization. The densitometric evaluation of protein bands was performed; when multiple bands for a protein were present, they were considered together in the densitometric evaluation. The numbers at the bottom of the Western blots indicate the fold variations for pTwist1/Twist and pWwox/Wwox ratios after HGF or TGFβ1 treatment versus the corresponding value of starved cells, considered as 1. The graphics in **a** and **c** show the changes of protein levels after the treatments, and the data are the means ± S.E. of three independent experiments. Where the S.E. bars are not shown, they lie in the symbol. *P < 0.05, **P < 0.005 versus the starvation value (Δ)

In cytosolic extracts (Fig. 1c), HGF progressively increased Twist protein level, which appeared phosphorylated mostly at 1 h diminishing thereafter. In contrast, TGFβ1 persistently enhanced Snail starting from 4 h, while progressively reduced pTwist1/Twist ratio. HGF and TGFβ1 augmented Wwox phosphorylation at 24 and 4 h, respectively.

The data show different effects of HGF and TGFβ1 on Twist and Snail patterns in nuclei, important for their transcription factor activity [7], and also differences in the relationship with Wwox phosphorylation. HGF caused early Twist1 phosphorylation and access to nuclei, while at later times Twist exit from the nucleus into the cytosol seemed to be preceded by nuclear-Wwox phosphorylation. Under TGFβ1, however, phosphoWwox and Snail were present concomitantly in the nucleus.

Further experiments were performed to clarify the molecular mechanisms of nuclear localization and function of Twist and its phosphorylation in response to HGF, by considering the involvement of Akt activity and the role of endogenous or exogenous Wwox on Twist activity (Fig. 2).

**Fig. 2:** Regulation of phosphoTwist1 nuclear localization and of Twist activity. In **a** and **b** we show representative images of Western blots, performed with nuclear, cytosol and total protein extracts of treated cells. The experiments were repeated three times with similar results. The samples were run on gel, and were processed under the same experimental conditions. B23 and vinculin were used for normalization. The numbers at the bottom indicate the fold variations for **a** pTwist1/Twist ratio and for **b** pAkt/Akt ratio versus the respective value of starved cells, considered as 1. **c** The cells were transiently transfected with Twist-gene reporter (TwistLuc), and co-transfected with siRNAWWOX or siRNAcontrol in the presence or the absence of *WWOX*-expression vector (e.v.). The histograms indicate the absolute values of Firefly/*Renilla* luciferase activity ratios. The data are the means ± S.E. of three independent experiments performed in triplicate. **P < 0.005, ***P < 0.001 versus TwistLuc-basal value (first bar); ^Δ^ *P* < 0.05 versus the luciferase activity in the presence of siRNAWWOX alone; ^○○^ *P* < 0.005 versus the luciferase activity value in the presence of siRNAcontrol plus *WWOX* e.v. Under these experimental conditions, we also show the Western blots of Wwox, Twist and pTwist1, and the experiments were repeated three times with similar results. The cytosolic and nuclear protein samples were run on gel, and were processed under the same experimental conditions. Vinculin and B23 were used for normalization. The numbers at the bottom indicate the fold variations relative to the siRNA control value, considered as 1. **d** The histograms indicate the fold changes of Wwox protein levels evaluated by Western blot. The normalization was performed with vinculin. The data are the means ± S.E. of three experiments. ***P < 0.001 versus basal value, considered as 1; ^○○^ *P* < 0.005 versus the value in the presence of *WWOX* e.v. **e** The cells were transiently transfected with TwistLuc, were co-transfected with *WWOX* e.v. or siRNAWWOX, were starved and were exposed to HGF. The histograms indicate the absolute values of Firefly/*Renilla* luciferase activity ratios. The data are the means ± S.E. of three independent experiments performed in triplicate. **P < 0.005, versus TwistLuc-basal value (first bar); ^Δ^ *P* < 0.05 versus the luciferase activity in the presence of HGF

Twist1 phosphorylation by Akt was studied using LY294002, a specific inhibitor of PI3K/Akt pathway, since Akt is stimulated by HGF in 1833 cells [25] and it is known to activate Twist in metastasis [28]. As shown in Fig. 2a, in nucleus and cytosol the phosphoTwist1 enhancements after 1-h HGF were prevented by LY294002. We showed that LY294002 inhibited Akt phosphorylation, index of its activity, under our experimental conditions (Fig. 2b).

Since HGF down-regulated nuclear Wwox, we evaluated the effect of siRNAWWOX on Twist activity. Figure 2c shows that siRNAWWOX increased TwistLuc activity in respect to untransfected (c) and siRNAcontrol-transfected cells. In contrast, *WWOX* expression vector (e.v.) reduced Twist-luciferase activity in untransfected, siRNAcontrol- and siRNAWWOX-transfected cells. The data of Western blots gave an explanation, because siRNAWWOX transfection largely reduced Wwox-protein levels in cytosol and nuclei, while *WWOX* e.v. co-transfection caused Wwox-protein accumulation in the cytosol, much more than in nuclei. siRNAWWOX reduced (−70 %) the protein level of Wwox under expression vector co-transfection (Fig. 2d).

As shown in Fig. 2e, the separate transfection of siRNAWWOX and *WWOX* e.v. oppositely affected TwistLuc, and overexpression of Wwox almost completely prevented HGF-dependent luciferase activation.

Altogether, the high-cytosolic Wwox seemed related to Twist-transactivation decrease, opposite to Wwox depletion being stimulatory for TwistLuc. The nuclear depletion of Wwox was, indeed, correlated with Twist1 access to the nucleus in the phosphorylated form, while Wwox overexpression augmented cytosolic-unphosphorylated Twist. Therefore, Wwox levels might participate in the nuclear phosphoTwist1 translocation and function.

### The intracellular distribution of Twist and Snail at early and later times after HGF differed depending also on the regulation exerted by HGF on TGFβ signalling

Figure 3a reports that HGF between 4 and 16 h strongly enhanced nuclear Twist and that, thereafter, the signal diffused to all the cell, as shown at 24 h. Under 4-h HGF, *WWOX* e.v. and siRNAWWOX caused Twist accumulation in the cytosol and in the nuclei, respectively (Fig. 3a, left panels). The transfection of siRNA control did not affect Twist distribution due to HGF (data not shown). Additional file 1: Figure S1 reports cellular Wwox distribution under the above reported experimental conditions. Figure 3a also shows that the cellular Snail slightly and progressively augmented under HGF, but it was strongly enhanced by TGFβ1 starting from 4 h until the end of the observation period. Cellular Twist slightly increased at later times after TGFβ1. After 4-h HGF, nuclear phosphoTwist1 signal was found (Fig. 3b).

**Figure 3:** Twist and Snail distribution in 1833 cells in response to HGF and TGFβ signallings. **a** The cells were exposed to HGF or TGFβ1 for various times on coverslips, with or without *WWOX* e.v. or siRNAWWOX, and were probed with anti-Twist (*green*) or anti-Snail (*red*) antibody. The nuclei were stained with DAPI (*blue*). The panels 1, 2, 3 show the merge images: 1 = green/DAPI; 2 = red/DAPI; 3 = green/red. **b** The cells exposed to 4-h HGF on coverslips, were probed with anti-pTwist1 (*magenta*) antibody; the nuclei were stained with DAPI, and their merge images are shown. For **a** and **b** the images, taken at 400× magnification, are representative of experiments performed in triplicate. **c** Representative images of Western blots repeated three times are shown, and the phosphoAMPK/AMPK ratio is indicated. The ratios were calculated using the densitometric values, obtained by taking into consideration all the specific-protein bands in each lane. Vinculin was used for normalization. **d** The cells, transfected with the 3TPLux gene reporter, were exposed to HGF in the presence or the absence of Compound C. The data are the means ± S.E. of three independent experiments performed in triplicate. ***P < 0.001 versus basal luciferase activity; ^ΔΔΔ^ *P* < 0.001 versus the luciferase activity under HGF

Thus, in response to HGF and TGFβ1, protein levels and intracellular localization of Twist and Snail were consistent with the distribution of their signals observed by immunofluorescence. Of note, the 1833 cells exposed to HGF for 24 h had a morphology more elongated (mesenchymal)- with preponderant Snail- than 1833 cells at early times after HGF, that seemed epithelial and clustered showing nuclear Twist. This might be index of Twist program activation. Also, the data led to hypothesize that HGF regulated TGFβ signalling, since Snail is a TGFβ-target gene [29], and suggested to study the gene patterns typical of EMT and MET under the two microenvironment stimuli. These studies were performed in invasive parental MDA-MB231 breast carcinoma cells and the derived 1833-bone metastatic clone. The comparative study of transcriptomic profile of the two cell lines identifies a gene set whose expression is associated with, and promotes the formation of metastasis to bone [20]. MDA-MB231 cells are invasive, and when metastasize they have tropism for various organs, and give metastasis to bone less efficiently and more slowly than 1833 cells [2].

First, we studied the role of AMPK under HGF on the luciferase activity of 3TPLux, a construct containing a strong TGFβ-responsive element that is routinely used to assay TGFβ signalling [30]. In other cell systems, AMPK is involved in HGF-TGFβ reciprocal regulation [31]. In 1833 cells exposed to HGF, AMPK phosphorylation progressively increased starting from 0.5 h, reaching the maximal values between 16 and 24 h (Fig. 3c). Moreover, we found that HGF increased 3TPLux activity (about 6-fold), and that the specific AMPK blockade with Compound C almost completely prevented the HGF-dependent luciferase activation (Fig. 3d). Additional file 2: Figure S2 shows 3TPLux activity in MDA-MB231 cells, also under AMPK blockade with Compound C.

### Effects of HGF and TGFβ1 on gene patterns of 1833 and MDA-MB231 cells, and on E-cadherin transactivation

Next, experiments were performed dealing with HGF and TGFβ1 involvement in MET versus EMT, by examining the patterns of the principal genes responsible for these phenotypes (Fig. 4).

**Figure 4:** HGF and TGFβ1 oppositely influenced the patterns of MET/EMT genes in 1833 and MDA-MB231 cells. **a**, **b** and **c** Representative images of Western blots performed with total protein extracts from 1833 and MDA-MB231 cells. The experiments were repeated three times with similar results. The samples were run on gel, and were processed under the same experimental conditions. Vinculin was used for normalization. For **a** and **b**, the numbers at the bottom indicate the fold variations relative to the starvation value, considered as 1; for **c**, the E-cadherin value for MDA-MB231 cells was compared to that of 1833 cells. For MMP2, the fold variations were calculated for the active form. **d** The cells, exposed to 1-h HGF on coverslips, were probed with anti-E-cadherin antibody (*red*); the nuclei were stained with DAPI, and their merge images are shown. All the images, taken at 400× magnification, are representative of experiments performed in triplicate. **e** Transcription-factor binding sites present in the entire E-cadherin promoter are shown. The 1833 cells, transiently transfected with the construct containing the entire E-cadherin promoter, were co-transfected with Twist-dominant negative (ΔTwist), WWOX e.v. or siRNAWWOX in the presence or the absence of HGF and TGFβ1. The histograms indicate the absolute values of Firefly/*Renilla* luciferase activity ratios. The data are the means ± S.E. of three independent experiments performed in triplicate. *P < 0.05, **P < 0.005 versus the basal luciferase activity value; ^Δ^ *P* < 0.05, ^ΔΔ^ *P* < 0.005 versus the luciferase activity value in response to HGF

In HGF-treated 1833 cells (Fig. 4a), E-cadherin increased early, peaking at 1 h and remaining elevated thereafter, with a return to the starvation value at 24 h, while protein levels of vimentin and MMP2 suddenly dropped almost disappearing from 6 h until the end of the observation period: the patterns of the three markers indicated prevalent MET transition. In contrast, TGFβ1 induced N-cadherin, vimentin and MMP2-active form, with MMP2-precursor (pro72) degradation contributing to the increase in the active form, while E-cadherin progressively decreased after TGFβ1 (Fig. 4a). As shown in Fig. 4b, the EMT markers Snail and vimentin were expressed in MDA-MB231 cells and were further augmented by TGFβ1, while HGF was ineffective; Twist1 phosphorylation was scarce, undergoing slight down-regulation under the two stimuli. Wwox-protein level, extremely low in MDA-MB231 compared to 1833 cells in agreement with previous data [19], was unaffected by HGF and TGFβ1. As shown in Additional file 2: Figure S2, HGF effect was studied on Twist transactivating activity in MDA-MB231 cells under HGF. Since Wwox did not seem present in this cell line, we did not study siRNAWWOX effect.

Taking into consideration all the data in 1833 cells, the return of E-cadherin to basal value 24 h after HGF might contribute to their reversion to a mesenchymal phenotype, consistent with immunofluorescence data; since HGF and TGFβ1 oppositely affected MET and EMT markers including E-cadherin, as reported for Twist, the latter might be differently involved in E-cadherin expression under the two biological stimuli. The regulation of E-cadherin deserves further attention.

Figure 4c shows that E-cadherin was expressed in 1833 clone but was practically absent in MDA-MB231 cells, as previously reported [19]. In 1833 cells, E-cadherin localized at plasma-membrane level, and increased under HGF; the merge showed a slight signal also in nuclei (Fig. 4d).

Experiments on E-cadherin transactivation in 1833 cells were performed under the two environmental stimuli to evaluate the role of Twist and Wwox, by transfecting the construct containing the entire E-cadherin promoter (Fig. 4e). The putative consensus sequences, present in the entire E-cadherin promoter and in the ΔPPRE-promoter fragment are shown. E-cadherinLuc was activated 4.5-fold by HGF, but was unaffected by TGFβ1. Twist seemed involved in the luciferase activation, because ΔTwist prevented of 40 and 60 % basal and HGF-stimulated E-cadherinLuc activity, respectively. *WWOX* e.v. reduced basal and HGF-induced E-cadherinLuc activity, while siRNAWWOX enhanced basal luciferase activity. All these data supported the role of Twist and Wwox in E-cadherin transactivation.

### Deepening of the role of transcription factors involved in E-cadherin transactivation under HGF and TGFβ1

Under HGF and TGFβ1, we evaluated the activities of the transcription factors presenting numerous-consensus sequences in the E-cadherin promoter, considering the function played by Twist. As shown in Fig. 5a and b, we started to clarify the involvement of PPARγ transcription factor in E-cadherin transactivation using ECad-LucΔPPRE gene reporter, i.e., the fragment lacking PPARγ-consensus site (PPRE) and the upstream sequence, and the construct containing the PPRE multimer (PPARγLuc). Then, the activities of the gene reporters driven by Ets1 or NF-*k*B multimers were evaluated (Fig. 5b). HGF enhanced E-cadherinLuc ΔPPRE activity, even if at a lesser extent in respect to the entire promoter, and ΔTwist partially prevented (30 %) this stimulatory effect (Fig. 5a). HGF activated PPARγLuc, Ets1Luc and NFkBLuc, while TGFβ1 activated only PPARγLuc. Twist was involved in all the luciferases activated by HGF, especially in PPARγLuc and Ets1Luc, as demonstrated with ΔTwist (Fig. 5b).

**Fig. 5:** Twist played a specific role in E-cadherin transactivation stimulated by HGF through PPARγ/Ets1/NF-*k*B activities. **a**, **b**, **c**, **d** and **e** The 1833 cells, transiently transfected with the E-cadherin promoter-ΔPPRE fragment, the various constructs containing the gene reporter driven by transcription-factor multimer, E-cadherin short fragments wild type (ECad-wtLuc) and E-boxes-mutated (ECad-mutLuc), or the entire E-cadherin promoter (ECadLuc), were co-transfected with ΔTwist or ΔARNT in the presence or the absence of HGF and TGFβ1. ECad-wtLuc and ECad-mutLuc structures are shown. The histograms indicate the absolute values of Firefly/*Renilla* luciferase activity ratios. The data are the means ± S.E. of three independent experiments performed in triplicate. *P < 0.05, **P < 0.005 versus the respective basal luciferase activity; ^Δ^ *P* < 0.05, ^ΔΔ^ *P* < 0.005 versus the respective luciferase activity in response to HGF

Other regulatory mechanisms for E-cadherin transactivation were investigated, because the E-cadherin promoter also contains 3 E-boxes (see Scheme Fig. 5c), and 8 HIF-1 consensus sites (HRE). Since the candidate target genes of Twist are analyzed for containing conserved E-box sequences [26], the activation of the wild-type short promoter fragment of E-cadherin under HGF, if any occurs, might indicate Twist functionality through E-boxes. In 1833 cells, HGF did not affect E-cadherin-luciferase activity of both wild-type and mutated short promoters (Fig. 5c).

Considering all the data, Twist seemed implicated in E-cadherin induction through the activation of PPARγ/Ets1/NF-*k*B transcription-factor network.

Notwithstanding HGF diminished (−50 %) HRELuc activity (Fig. 5d), we examined the effect of the dominant negative of HIF-1β subunit (ΔARNT) on E-cadherin transactivation by HGF (Fig. 5e). ΔARNT prevented the stimulation of the E-cadherin luciferase activity by HGF, suggesting that HIF-1 activity was implicated in HGF-dependent E-cadherin induction only within a network of transcription factors and/or co-factors cooperating on gene promoter. For example, a cooperative function of Wwox and Twist might occur.

To better understand HIF-1-activity regulation under our experimental conditions, we evaluated the effect of exogenous Wwox, and the role played by Twist (Fig. 6). *WWOX* e.v. enhanced the protein levels of Twist, Snail and Wwox itself (Fig. 6a). As shown in Fig. 6b, exogenous Wwox tripled HRELuc, that was completely prevented by ΔTwist; basal HRELuc activity was also diminished by ΔTwist. The implication of Twist in HIF-1 activity was corroborated by gel shift and super-gel shift experiments, using an oligonucleotide sequence present in E-cadherin promoter that contains 1 HRE (Fig. 6c). The transfection of *WWOX* e.v. increased the specific DNA binding of the HIF-1 dimer, and the constitutive binding. The presence of the HIF-1α subunit in the DNA bindings was verified by a super-gel shift experiment, using anti-HIF-1α antibody that gave immunodepletion, consistent with previous data obtained in 1833 cells with the same oligonucleotide [32]. Interestingly, anti-Twist antibody also gave immunodepletion of specific and constitutive bindings, indicating Twist as co-factor of HIF-1 under Wwox overexpression. The specificity of the findings was demonstrated as follows: anti-Ets1 antibody did not affect the HIF-1-DNA binding in response to *WWOX* e.v, and the specific competition reduced the specific binding (Fig. 6c).

**Fig. 6:** HIF-1 transactivating activity and its DNA binding, and TGFβ1 transactivating activity under *WWOX* expression vector. **a** Representative images of Western blots repeated three times are shown. Vinculin was used for normalization. The numbers at the bottom indicate the fold variations relative to control, considered as 1. **b** The cells, transfected with the gene reporter driven by the HRE multimer, were co-transfected with *WWOX* e.v. in the presence of the absence of ΔTwist. The data are the means ± S.E. of three independent experiments performed in triplicate. *P < 0.05, **P < 0.005 versus basal luciferase activity; ^ΔΔΔ^ *P* < 0.001 versus luciferase activity under *WWOX* e.v. **c** Nuclear extracts from control or *WWOX* e.v.-transfected cells were used for DNA-binding assay, and super-gelshift with the indicated antibodies was done. 50× competition was performed with an excess of unlabeled oligonucleotide. const, constitutive binding. A representative image of three independent experiments is reported. **d** The cells, transfected with the construct containing the entire TGFβ1 promoter or its fragment (see Scheme), were co-transfected with *WWOX* e.v. in the presence or the absence of ΔTwist. The data are the means ± S.E. of three independent experiments performed in triplicate. **P < 0.005, ***P < 0.001 versus respective basal luciferase activity; ^Δ^ *P* < 0.05 versus the luciferase activity in response to *WWOX* e.v.; °*P* < 0.05 versus the luciferase activity in the presence of ΔTwist

The activity of TGFβ1 promoter was also studied because it contains 1 USF1/2 (E-box) sequence and 5 HRE sites [33, 34], leading to hypothesize that TGFβ1 is a target gene of Twist. The TGFβ1-promoter fragment lacking the USF1/2 (E-box) sequence, shows only one HRE (Fig. 6d). *WWOX* e.v. was ineffective on the luciferase activity of the two constructs, while ΔTwist exerted an inhibitory effect on TGFβLuc, independent on E-box sequences, suggesting that Twist implication in basal luciferase activity did not require E-box regulation. Wwox overexpression was additive with ΔTwist in inhibiting TGFβLuc of the entire promoter, possibly due to the interference with HIF-1 binding to HRE. In fact, using the TGFβLuc fragment, *WWOX* e.v. partially prevented the inhibitory effect.

The data show that HGF, reducing nuclear-protein level of Wwox, and *WWOX* e.v., increasing Wwox protein level, had opposite effects on HIF-1 transactivating activity.

## Discussion

MET has been proposed as the phenotype acquired by breast cancer for establishment of metastases in adjacent-lymphovascular space [35], lung [12] and skeleton [19]. For bone metastasis, however, exhaustive experimental evidence is still lacking, that would clarify the involvement of microenvironmental stimuli and the underlying molecular and signalling events. Here, we show a key role of HGF, a paracrine-biological stimulus of bone pre-metastatic niche, in determining MET gene profile important for the colonization of breast cancer metastasis to bone. In fact, HGF-dependent MET switch occurred through Twist-program activation, even if this process was transient. HGF regulated TGFβ signalling and the transcriptional network downstream in a time-dependent manner, conferring phenotype plasticity to bone metastasis with the return to EMT. Noteworthy, Twist and Snail were differently responsive to the two biological stimuli through Wwox changes, regulating in bone metastasis non-redundant pathways.

First, we discuss in bone metastatic cells the critical role played by HGF in the triggering of Twist program, and its functional significance, at a difference with TGFβ1. HGF dictated Twist expression and phosphorylation in 1833 cells, and PI3K/Akt signalling pathway was responsible for the phosphorylation in Ser42 of Twist1. PhosphoTwist1 presence in nuclei, that might depend on the decrease of Wwox, played an important role in mediating PPARγ/Ets1/NF-*k*B-dependent induction of E-cadherin under HGF. The slowing down of HGF-dependent stimulatory effect on Twist program, due to nucleo-cytoplasmic shuttle of Twist, seemed to be due to nuclear phosphorylation of Wwox with cytosolic accumulation of unphosphorylated Twist. Our findings agreed with Twist1 expression in bone metastasis formation, and with phosphoTwist controlling the interaction with distinct transcription factors [27, 28].

Altogether, the cross-talk with gene regulators like Wwox, but not E-box-regulation, was an important mechanism by which Twist mediated E-cadherin transactivation in 1833 cells exposed to HGF, in agreement with the fact that bHLH function depends on protein-protein interactions [36]. In normal mammary epithelial cells, Twist1 induces dissemination without loss of epithelial gene expression and requires E-cadherin [37], consistent with our data in metastatic cells in which Twist program positively influenced the adhesive properties and MET phenotype. In particular, Wwox-knocking down increased Twist access to nuclei and its activity. In contrast, Wwox overexpression counteracted the stimulatory effect of HGF on Twist access to nuclei and Twist transactivating activity preventing E-cadherin induction. The transcriptional pattern downstream of HGF seemed to depend on the cell type, and we cannot exclude that the specific pattern of HGF signalling via Twist was related to E-cadherin induction. In fact, in MDA-MB231 breast carcinoma cells, that did not show E-cadherin, HGF was ineffective on Twist expression/transactivating activity and Snail expression, while in HepG2 hepatocarcinoma cells HGF induces upregulation of Snail through MAPK/Erg-1 pathway, without affecting Twist, leading to downregulation of E-cadherin [38]. It is likely that in 1833 cells, Snail could be activated indirectly by HGF consequent to the TGFβ-signalling induction. At later times after HGF, Snail signal was found in 1833 cells that switched to the mesenchymal phenotype.

We suggest the involvement of protein stabilization in the very rapid E-cadherin induction by HGF. The half-life of E-cadherin is approximately 5 to 10 h, and the transcriptional regulation cannot account for the most rapid changes in adhesion strength [39]. Endocytosis, degradation and recycling of E-cadherin are crucial for dynamic regulation of adherens junctions and for the control of intercellular adhesion. The E-cadherin expression/trafficking seemed differently regulated by HGF and TGFβ signals in 1833 cells. TGFβ1 down-regulated E-cadherin, and conferred the characteristic EMT-gene profile, comprising N-cadherin, vimentin, MMP2 and Snail expression. Snail is known to be implicated in E-cadherin down-regulation [9, 10, 38]. Moreover, TGFβ activates ERK2 that directly phosphorylates Snail, leading to its nuclear accumulation, reduced ubiquitination and increased protein half-life [29], while HGF is practically ineffective on ERK1/2 phosphorylation in 1833 cells [25]. As in HGF-treated 1833 cells, also in the xenograft model the bone-metastatic cascade invokes E-cadherin emergence [19], consistent with the MET process in response to HGF [2, 25].

Second, our findings suggest for Twist a complex spatio-temporal expression and function, also related to the composition of bHLH-dimer pool [26], with a critical role of Twist as HIF-1 co-activator under Wwox overexpression.

We found Wwox in bone-marrow supportive cells (Additional file 3: Figure S3), where it might influence metastatic-cell signalling profiles also regulating HIF-1 target genes [40]. Thus, exogenous *WWOX* might mimic the effects of this anomalous-tumour suppressor present in the microenvironment for the cross-talk with bone metastasis. Substantially differing from the molecular events triggered by endogenous Wwox, that was phosphorylated by growth factors, microenvironmental Wwox is supposed to interact with proteins in membrane-cytoskeleton area regulating acidic-secretion as ezrin [41], or to influence TFGβ binding to hyaluronan/hyaluronidase-Hyal-2 and its internalization [22]. Extracellular pH is tightly regulated within bone, and it has significant effects on osteoblast and osteoclast function [42].

Third, another worth noting aspect was the relationship of bone metastasis plasticity to the HGF-dependent activation of TGFβ signalling via AMPK activity. As consequence, a hierarchic response of Twist and Snail occurred. This intricate mechanism explains the *in vivo* data, since the reversion of MET to EMT phenotype might be important for colonization coupled to osteolysis [43]. In fact, Twist1 expression also regulates the activity of the osteoclasts in bone metastasis [27]. In the bone matrix, TGFβ is one of the most abundant growth factors, which is released in active form upon metastasis-induced bone resorption by osteoclasts, and which emerges as a potent driver of progression through its immunosuppressive, proangiogenic and EMT inducer roles [44, 45]. The MET inducing changes due to HGF were, therefore, transient in nature and did not involve permanent genetic-alterations in EMT regulators. We hypothesize that metastatic cells adopt a plastic phenotype in response to biological stimuli to overcome the different hurdles encountered. In this regard, inhibiting either EMT or MET alone may have unwanted adverse side effects, and the therapeutic window for applying EMT/MET targeting treatments needs to be carefully evaluated. Developing drugs that target particular phases of metastasis is of paramount importance. For example, targeting HGF of pre-metastatic niche would reduce Twist1 phosphorylation important for E-cadherin expression in bone metastasis colonization.

## Conclusions

The Scheme (Fig. 7) summarizes the molecular findings of the present paper on the stimulatory effect of HGF on Twist nuclear localization and Twist program. Twist activity and endogenous Wwox co-factor appeared to function along a common signalling pathway triggered by HGF (see Fig. 2e). Also, we suggest a relationship with the immunohistochemical data of E-cadherin in pair-matched primary-ductal breast carcinoma and bone metastasis from humans, where E-cadherin expression is absent and present, respectively [19]. HGF/Met system is elevated in bone metastasis [2, 25], and might cooperate also *in vivo* with TGFβ signalling [20], affecting the intercellular adhesive properties and colonization.

**Fig. 7:** Relationship of molecular data *in vitro* with E-cadherin immunohistochemistry in bone metastasis and primary-breast carcinoma. A schematic representation of the molecular data obtained with 1833 cells is reported as well as the relationship with E-cadherin immunohistochemistry data in bone metastasis (me) and primary breast carcinoma (ca). We analyzed samples from three different patients, using five serial sections for each specimen of me and ca, and representative images are shown. Negative controls were performed without the specific antibody. HGF seemed to play the principal role in E-cadherin induction through Twist-nuclear localization and activation of PPARγ/Ets1/NF-*k*B transcription factors, in agreement with MET phenotype and E-cadherin expression at plasma membrane level in metastasis. The molecular pattern consisted in HGF-dependent inhibition of the down-regulatory function of Wwox. In contrast, TGFβ might be involved in EMT without E-cadherin expression, as occurs in primary-breast carcinoma. One possible molecular mechanism seemed to be the activation of Snail, a target gene of TGFβ, that was involved in E-cadherin down-regulation. In 1833 cells, exogenous Wwox by enhancing Twist-HIF-1 interaction might be important for Snail inhibitory function on target genes [51]

## Methods

### Reagents and plasmids

Recombinant-human HGF and TGF-β1 were from R&D System (Abingdon, UK). For Western blots, anti-Twist1/2 (H-81), anti-Wwox (N-19), anti–N-cadherin (H-4), anti-AMPKα1/2 (H-300), anti-phosphoAMPKα (Thr 172), anti Akt1/2 (H-136), anti-Ets1 (C20) and anti-vimentin (V9) antibodies were from Santa Cruz-Biotechnology (Santa Cruz, CA, USA); anti-Snail 1/2 antibody (ab53519) and anti-phosphoWwox (phosphoY33) were from Abcam (Cambridge, UK); anti-E-cadherin (clone 36) was from Transduction Laboratories (Lexington, KY, USA); anti-MMP-2 and anti-phosphoAkt were from Cell Signaling Technology (Beverly, MA, USA); anti-phosphoTwist1 (Ser42) was a generous gift of B. Hemmings (Friedrich Mieschern Institute for Biomedical Research, Basel, Switzerland). Anti-HIF-1α antibody (OZ12) was from NeoMarkers-LabVision Co (Fremont, CA, USA). Anti-Wwox antibody for immunohistochemistry (IMG-4187) was from Imgenex (San Diego, CA, USA). Alexa Fluor 488, 568 and 647 were from Molecular Probes (Eugene, OR, USA). siRNAcontrol and siRNAWWOX were from Dharmacon (GE Healthcare, Milan, Italy). The expression vectors were: WWOX (S. Semba, Kobe University, Japan), Twist dominant negative (ΔTwist) (E-M. Füchtbauer, Aarhus University, Denmark), HIF-1β dominant negative (ΔARNT) (M. Schwarz, University of Tübingen, Germany). The gene reporters were: the entire E-cadherin (−3059/+298) promoter and its PPRE-lacking fragment (−2461/+298) (J. Teyssier, Inserm-Montpellier, France); the E-cadherin short promoters, wild-type and mutated in the three E-boxes (Addgene); PPRELuc, containing 3-PPRE consensus sequences (R.M. Evans, Salk Institute for Biological Studies, San Diego, CA); HRELuc, containing 6-Hypoxia responsive elements (HRE) (P.J. Ratcliffe, Welcome Trust Center for Human Genetics-Oxford, UK); the construct containing 5-Ets-1 consensus sequences [46]; the NFKBLuc containing 3-NFkB binding sites (M. Hung, Anderson Cancer Center, Huston, TX); the Twist promoter (TwistLuc), (M-C. Hung, University of Texas, USA); the entire TGFβ promoter (TGFβLuc, −1362/+11) and its fragment (−453/+11) (G. Waris, Rosalind Franklin University, Chicago, IL); 3TPLux (Addgene). LY294002 was from Calbiochem (Merk Millipore, Milan, Italy). Fugene 6 was from Roche Applied Science (Monza, Italy); Lipofectamine 2000 was from Invitrogen (Milan, Italy).

### Cell cultures and treatments

1833 bone-metastatic clone and the parental MDA-MB 231 cells in the year 2008 were furnished by R. Gomis’ laboratory (IRB, Barcelona, Spain), on behalf of J. Massaguè (Memorial Sloan-Kettering Cancer Center, New York, NY, USA). The method short tandem repeat profiling (STR) of nine highly polymorphic STR loci plus amelogenin was used to authenticate MDA-MB 231 and 1833 cells in September 2014 (Cell Service from IRCCS Azienda Ospedaliera Universitaria San Martino-IST-Istituto Nazionale per la Ricerca sul Cancro, Genova, Italy).

The cells, routinely maintained in DMEM containing 10 % (v/v) FBS, were used after 2 or 3 passages in culture. They were treated with recombinant-human HGF (100 ng/ml) or recombinant-human TGF-β1 (5 ng/ml) [47] after 24-h starvation. 20 μM LY294002 was added to the cells 30 min before HGF exposure [46]. The concentrations used for the growth factors *in vitro* were in the range of those observed for HGF and for TGFβ in the plasma of cancer patients [48, 49].

### Western blot analysis

Total and cytosol (100 μg of protein), and nuclear (50 μg of protein) extracts were examined by Western blot [24], and immunoblot was performed with anti-Twist (1:200), anti-phosphoTwist1 (1 μg/ml), anti-Snail 1/2 (1:500), anti-Wwox (1:200), anti-phosphoWwox (1:500), anti-E-cadherin (1:1000), anti-N-cadherin (1:300), anti-vimentin (1 μg/ml), anti-MMP2 (1:1000), anti-Akt (1:200), anti-phosphoAkt (1:1000), anti-AMPK (1 μg/ml) or anti-phosphoAMPK (1 μg/ml) antibody. Densitometric analysis was performed after reaction with ECL plus chemiluminescence kit from Thermo-Fisher Scientific (Waltham, MA, USA).

### Luciferase reporter assay

The cells in 24-multiwell plates at 70 to 80 % of confluence, were incubated with a mixture (3:1) of DNA and Fugene 6, containing the internal control pRL-TK (*Renilla* luciferase plasmid). Gene reporters and expression vectors (0.4 μg/ml), or the dominant negatives ΔTwist (1 μg/ml) and ΔARNT (2 μg/ml) were transfected for 24 h. Equivalent amounts of empty vectors were tested. All the expression vectors were transfected in proportion 1:5, in respect to the internal control. After starvation for 18 h, the transfected cells were exposed to HGF or TGFβ1 for further 24 h. After 18-h 3TPLux-transfection under starvation, we performed the 24-h treatment with HGF in the presence or the absence of 10 μM Compound C [50]. Firefly/*Renilla* luciferase activity ratios, calculated by the software, are reported as absolute values. siRNAWWOX and siRNAcontrol were transfected for 48 h with Lipofectamine 2000 [19].

### Immunofluorescence assay

1833 cells (4 × 10^4^) on coverslips were transfected with *WWOX* e.v. or siRNAWWOX, were starved, were exposed to HGF or TGFβ1 and were probed with the following antibodies: anti-Twist, anti-phosphoTwist1, anti-Snail antibody (1:50), anti-E-cadherin antibody (1:5000) or anti-Wwox (N-19) (1:50). Secondary reactions with fluorescent antibodies were performed [2]. The images were collected under Eclipse 80i-Nikon Fluorescence microscope.

### EMSA analysis

Nuclear extracts from *WWOX* transfected cells were used for gelshift and super-gelshift assays [32]. For super-gelshift, the extracts were pre-incubated with l μg of anti-HIF-1α or of anti-Twist antibody for 1 h at 4 ° C, or with l μg of anti-Ets1 antibody for 15 min at room temperature, followed by the incubation with the labelled oligonucleotide drawn on E-cadherin promoter and containing 1 HRE (5’-GGAATCAGAACCGTGCAGGTCCCAT-3’, −224 to −200). For competition experiments, 50-fold excess of specific unlabeled oligonucleotide was added to the samples.

### Xenograft model and Immunohistochemistry

Animal studies were performed in conformity with the institutional guidelines, in compliance with national and international laws and policies. 1833 cells (5 × 10^5^) were injected in the left ventricle of the hearts of nu/nu mice (n = 5). Bones were collected at 26 days from cell injection; they were fixed and decalcified, and three serial sections were immunostained with anti-Wwox (1:200) antibody. Also, we analyzed five serial sections of pair-matched human specimens from primary-invasive ductal breast carcinoma (positive for oestrogen and progesterone receptors and negative for HER2) (n = 3) and from bone metastasis (n = 3) (Istituto Ortopedico Galeazzi, Milano, Italy). All patients provided informed consent, in accordance with Declaration of Helsinki. The bone specimens were fixed and decalcified before the manipulations. The sections of specimens from carcinomas and from bone with metastases were immunostained with anti-E-cadherin (1:100) antibody [19].

### Statistical analysis

Densitometric and luciferase activity values were analyzed using ANOVA, with P < 0.05 considered significant. Differences from controls were evaluated on original experimental data.

## Additional files

Additional file 1: Figure S1. Evaluation by immunofluorescence of Wwox changes in 1833 cells. We observed that 4-h HGF reduced the signal of cellular Wwox, with depletion of the nuclear content, and the concomitant transfection of *WWOX* e.v. caused a strong accumulation of Wwox in the cytosol. Under HGF, siRNAWWOX downregulated the cellular signal of Wwox. The anti-Wwox antibody (N19) (1:50 dilution) from Santa Cruz was used. Additional file 2: Figure S2. Effects of HGF on TGFβ signalling and Twist transactivating activity in MDA-MB231 cells. To make a comparison with 1833-bone metastatic cells, the effect of HGF on Twist program in parental MDA-MB231 breast carcinoma cells was examined. We studied under HGF the activities of 3TPLux, in the presence or the absence of Compound C to inhibit AMPK activity, and of TwistLuc. We found that HGF treatment did not modify 3TPLux activity, while Compound C alone or in the presence of HGF stimulated the TGFβ signalling. Thus, we can suggest that AMPK downregulated the TGFβ signalling under basal conditions in MDA-MB231 cells at a difference with 1833 cells. AMPK is known to mimic the inhibitory effect of HGF on TGFβ1 signalling of myofibroblasts differentiating from tendon fibroblasts [31]. In addition, TwistLuc activity was unmodified by HGF, in agreement with the ineffectiveness of HGF on phosphoTwist/Twist ratio shown in Fig. 4b of the present paper. Additional file 3: Figure S3. Wwox expression in the bone metastatic tissue of the xenograft mice. We evaluated by immunohistochemistry the expression of Wwox in the bone metastasis and the bone marrow of the xenograft model, due to the possible role of microenvironment in influencing cellular signals. This experiment was performed to give a biological significance to the *in vitro* treatment with *WWOX* expression vector, that increased ectopic Wwox in bone metastatic cells. Wwox was markedly present in metastasis (me), as previously reported [19], and was also evidenced in bone-marrow cells (bm), mostly at perinuclear level. The images were taken at 4×, 20× and 100× magnifications, and represent experiments repeated on three serial sections for each specimen from 5 mice. bo, bone.

## Abbreviations

MET: Mesenchymal-epithelial transition
EMT: Epithelial-mesenchymal transition
HIF-1: Hypoxia inducible factor-1
TGFβ: Transforming growth factor-β
Wwox: WW-domain containing oxidoreductase
HGF: Hepatocyte growth factor
PPRE: PPARγ-consensus sequence
